RETRACTED

# Double graph correlation encryption based on hyperchaos

**DOI:** 10.1371/journal.pone.0291759

**Published:** 2023-09-28

**Authors:** Luoyin Feng, Jize Du, Chong Fu

**Affiliations:** 1 School of Computer Science and Engineering, Northeastern University, Shenyang, China; 2 School of Electrical Engineering and Computer Science, University of Missouri, Columbia, Missouri, United States of America; Jaramogi Oginga Odinga University of Science and Technology, KENYA

## Abstract

Preventing unauthorized access to sensitive data has always been one of the main concerns in the field of information security. Accordingly, various solutions have been proposed to meet this requirement, among which encryption can be considered as one of the first and most effective solutions. The continuous increase in the computational power of computers and the rapid development of artificial intelligence techniques have made many previous encryption solutions not secure enough to protect data. Therefore, there is always a need to provide new and more efficient strategies for encrypting information. In this article, a two-way approach for information encryption based on chaos theory is presented. To this end, a new chaos model is first proposed. This model, in addition to having a larger key space and high sensitivity to slight key changes, can demonstrate a higher level of chaotic behavior compared to previous models. In the proposed method, first, the input is converted to a vector of bytes and first diffusion is applied on it. Then, the permutation order of chaotic sequence is used for diffusing bytes of data. In the next step, the chaotic sequence is used for applying second diffusion on confused data. Finally, to further reduce the data correlation, an iterative reversible rule-based model is used to apply final diffusion on data. The performance of the proposed method in encrypting image, text, and audio data was evaluated. The analysis of the test results showed that the proposed encryption strategy can demonstrate a pattern close to a random state by reducing data correlation at least 28.57% compared to previous works. Also, the data encrypted by proposed method, show at least 14.15% and 1.79% increment in terms of MSE and BER, respectively. In addition, key sensitivity of 10^−28^ and average entropy of 7.9993 in the proposed model, indicate its high resistance to brute-force, statistical, plaintext and differential attacks.

## 1. Introduction

The protection of sensitive information from unauthorized access has been a concern for centuries. For this reason, methods of information encryption have been used even before the advent of computers, using simple techniques such as letter substitution for this purpose [1]. With the widespread use of computers, information encryption has entered a new phase, and complex and secure methods have been developed to protect information. The development of computer networks and the high volume of information exchanged through them has made efficient information encryption a more serious requirement than ever before. And as internet penetration and computer technologies increase in everyday life, this need becomes more urgent [2]. For this reason, we have seen various methods of encryption over the years. Each of these studies has tried to address the deficiencies of previous methods based on existing security concerns and threats. Despite the acceptable performance of existing encryption techniques, they cannot be considered as a final solution for encrypting all types of information. On the one hand, the exponential increase in computing power makes it easier for attackers to detect secret keys than before, and on the other hand, existing encryption methods do not perform equally well for different types of data [3]. For example, image encryption is different from text encryption due to some inherent features of images, such as the high volume of data and the high correlation between pixels, and classical text encryption methods are not very efficient for this purpose [4]. Therefore, providing efficient systems for encrypting various data types is always considered as one of the challenges of cryptography research, and among these encryption algorithms, image encryption has the largest share in the research conducted in the field of cryptography. Because image encryption techniques generally have a high ability to encrypt other types of data as well; But the reverse of this process is not necessarily true [5]. Thus, the need to provide efficient strategies for encryption of all types of information and with the ability to deal with existing security threats is always felt. Chaotic models are among the most widely used strategies for information encryption. Chaos-based encryption technique has several main features such as sensitivity to initial conditions, decisiveness and originality [6] and these features have led us to witness many encryption methods based on this solution in recent years. Nevertheless, one of the shortcomings of methods based on chaotic systems is the limited key space compared to other strategies, which can be effective in the vulnerability of the method against brute-force attacks [7]. In this article, a new strategy based on hyperchaos system is presented in order to solve the existing inadequacies. The contribution of the current article is as follows:

- In this article, a new chaotic model with high key space and also high key sensitivity is proposed, which eliminates the limitations related to the data types that can be encrypted in previous chaotic models.
- The proposed encryption solution in this article uses diffusion and confusion stages to enhance the information security level and can meet Shannon’s theoretical criteria.
- The proposed method in this article has been investigated against a wide range of visual attacks, correlation analysis, differential attacks, key sensitivity and time analysis to study the performance of the encryption system in terms of efficiency, stability, and resistance against analytical attacks.
- In this article, a rule-based reversible model is used to re-diffuse the data, which can minimize the correlation between the data in a way that the possibility of extracting the pattern of the relationship between the data is minimized.

RETRACTED

This article is organized as follows: In section two, the research background is reviewed and in section three, the proposed method for image encryption is presented. In section four, the results of implementing and evaluating the proposed encryption algorithm are presented, and in section five, the obtained results are discussed. Finally, some suggestions for further research are presented.

## 2. Related works

In recent years, the number of studies carried out in the field of encryption has been significant, indicating the importance of encryption and the need for new solutions to address the shortcomings of existing methods. In this section, we will focus on the study of some chaotic-based encryption techniques, based on the tools used in the research.

In [8], a substitution model and chaotic system are used to improve the efficiency of chaotic encryption systems. This method consists of four stages: initial diffusion, confusion, secondary diffusion, and final permutation. These stages are implemented by advanced chaotic map, S-Box, logistic map, and substitution function, respectively. The key space of the chaotic map used in this research is very limited which makes it vulnerable to exhaustive attacks. In [9], a combination of two-dimensional sinusoidal map and repeated chaotic map with infinite modulation is used to improve the key space. In this method, confusion and diffusion processes are combined in one step to reduce computation time. But this operation leads to relatively high correlation in encrypted images.

In [10], the authors design a four-dimensional discrete chaotic map using a linear balanced sine function for data encryption. The key space created by the chaotic map is greater than 2^1170^. This method provides a significant chaotic effect compared to other encryption techniques. However, the researchers have mostly focused on the analysis of key space and did not provide any information about histogram analysis, correlation analysis, entropy, etc. The research in [11] uses the concept of data filtering in encryption to increase data security. This method is suitable for encryption applications where data integrity is not a priority, as filtering can spread small changes in plain data to all encrypted data bytes. This method provides better results than its previous encryption techniques in terms of statistical and differential attacks. The method presented in [12] introduces a new chaotic system by the difference of output sequences of two similar chaotic systems, which addresses the flaws of a single map. Data encryption in this method is performed during the processes of confusion, diffusion, and re-confusion. However, the authors did not discuss the efficiency of this encryption method against known-plaintext attacks.

RETRACTED

Research in [13], introduced a chaos based image encryption algorithm. In this method, the image is divided into several blocks and then, correlation coefficient (CC) of each block is calculated. This algorithm uses a Skewtent map to modify pixel values of blocks with higher CC and uses a static threshold of 0.3 for recognizing these blocks. Finally, a Tangent Delay Ellipse Reflecting Cavity Map System (TD-ERCS) map is used for permuting all blocks and producing encryption result. The Skewtent map used in this research does not reflect an appropriate chaotic behavior. This, results to high CC and low entropy of encrypted data.

In [14], a selective encryption algorithm using dual chaotic map and DeoxyriboNucleic Acid (DNA) rules which is suitable for medical images. This algorithm, applies confusion and diffusion operations on a selected subset of pixels. Then uses DNA rules to modify all pixels of the image. This research, reports low entropy and key sensitivity which makes it unsuitable for general applications. A similar research in [15], utilized combination of DNA rules and hyperchaotic maps to encrypt images. This algorithm, uses two rounds of diffusion for modifying pixels and generating DNA encoding rules based on the values of the pixels. Using pixels values as the seeds of rule generator makes this algorithm prone to error and very irritable against noise.

Research in [16], used chaos theory and wavelet decomposition approaches for image encryption. In this method, the input image is diffused by logistic map and chaotic transformation operator. Then, the diffused image is decomposed using continuous and discrete wavelet transform; followed by confusing each component of the decomposed image using chaotic transformation operator. Finally, the image is reconstructed using inverse continuous and discrete wavelet transform. Histograms of the encrypted images still reflect some parts of the histogram of the original image which makes this method vulnerable against statistical attacks.

RETRACTED

In [17], a multiple encryption algorithm for images is proposed using chaotic maps and wavelet transform. This method provides high security with low computation costs and is suitable for image encryption. In [18], a combination of Discrete FRactional Wavelet Transform (DFRWT) and quantum chaos was used to encrypt images. In this method, a multi-scale decomposition of the original image is created using DFRWT. Then, the high and low frequency coefficients in the time-frequency-domain are permuted, and the inverse DFRWT is applied to the image to produce the resulting encryption. Finally, using the XOR operator, the permuted sequence and quantum chaotic sequence are combined to produce the encrypted data. Methods [17, 18] cause partial changes in the decrypted images and are not suitable for applications which data integrity is important.

In [19], a chaotic-based encryption method is proposed. The chaotic model defined in this study uses three keys, and a substitution matrix is used to generate their initial values. The algorithm is formulated using the Fiestel network and some of the Advanced Encryption Standard (AES) encryption steps. The AES mechanism in this algorithm, consumes a relatively high memory and processing power. In [20], a method for multi-image encryption using the chaotic systems and gene fusion is presented. In this method, the pixels of the images are permuted using a chaotic sequence, and then the pixels are rotated in a circular pattern. Next, a DNA rule controller is used to determine the encoding and decoding rules, which is also based on a chaotic system. Finally, the propagation process is performed on the group of images using gene fusion strategy to obtain the final encrypted image. The map used in this research, shows a chaotic behavior within a small range of secret key and is vulnerable to reconstruction. Also, the encryption time of this algorithm is relatively high.

In [21], an n-dimensional chaotic model based on the general Hamiltonian system is proposed. The n-dimensional model can address the limitations of basic chaotic models in terms of vulnerability to reconstruction. In this study, a 4-dimensional chaotic model is presented based on the proposed solution and then used for image encryption. In [22], a method based on block permutation and chaotic models is presented for encrypting color images. In this method, the image is first decomposed into R, G, and B color layers and then divided into blocks. Next, the pixels of each block are permuted, and then the blocks of the image are moved. Finally, a logistic map is used to change the pixel values of the permuted image. In this method, the colored layers of the encrypted images are highly correlated which their extracted information can be used as a tool for statistical attacks.

RETRACTED

In [23], a fractional-order chaotic system based on Hopfield Neural Networks (HNN) is first proposed, and then its application in image encryption is evaluated. In this study, the Adomain decomposition method is used to solve the proposed chaotic system. By changing its orders, this chaotic system can exhibit dynamic and chaotic behavior, and based on the pseudo-random numbers generated by it, a new method is proposed for constructing multi-chain hash indices. The method presented in [24] uses a combination of a chaotic model and a Kernel Auto‐Associated (KAA) map to encrypt color images. The model performs encryption based on two keys. The first key is generated based on a sinusoidal logistic map and a homogeneous linear generator, while the second key is created using a Tent map and a Bernoulli map. Finally, the diffusion process is carried out based on the KAA map. The encryption/decryption time for the methods of [23] and [24], are relatively high.

## 3. Research methodology

In this section, the details of the proposed encryption algorithm are described. To this end, a novel hyperchaotic model is introduced, and then the encryption stages of the proposed algorithm based on this model are presented.

### 3–1. Proposed chaotic model

A system with chaotic behavior that has at least two positive Lyapunov exponents is called a hyperchaotic system. Considering a void negative exponent along the sequence and a negative exponent to ensure the boundedness of the system, the minimum number of dimensions for a continuous hyperchaotic system is equal to 4. The Hénon map is one of the most well-known discrete chaoṁtic systems that maps a point such as (*x*_*n*_,*y*_*n*_)ṁ to a new point on the plane [26].


$$\left\{\begin{array}{l} x_{n+1}=1-\alpha x_{n}^{2}+y_{n}\\ y_{n+1}=\beta x_{n} \end{array}\right.$$ (1)

This hyperchaotic map is dependent on two parameters, α and β. A change in the values of these two parameters can result in chaotic behavior of the system. In Fig 1, the structure of the chaotic map obtained from Eq (1) based on the values of the two parameters α and β is shown. In this figure, the range of variation of the two parameters α and β is considered as 1 ≤ *α* ≤ 2 and 1.5 ≤ *β* ≤ 2 and the initial value *x*_0_ = 0.1 is assumed.

RETRACTED

**Fig 1:** Structure of the hyperchaotic map obtained from Eq (1) based on the values of the α and β keys.

As can be seen in Fig 1, if the two parameters α and β are in the range [1.55, 2.05], Eq (1) will exhibit chaotic behavior. However, this hyperchaotic map is faced with two fundamental problems that make its use for encryption applications difficult: Firstly, the key space in this system is very limited. Secondly, the sensitivity of each key is limited to 10^−10^. This means that using two keys with a difference of less than 10^−10^ will result in sequences that are almost identical. To overcome the limitations mentioned in this chaotic model, spatiotemporal-based systems can be used.

CML is a model that simulates a dynamic system with discrete space and position, which has sequential states and is often used as a primary model for studying the dynamics in chaotic space-time systems. A two-way CML system can be modeled as the following equation [27]:

$$\left\{\begin{array}{l} x_{n+1}=(1-\varepsilon )f\left(x_{n}(i)\right)+\frac{\varepsilon }{2}\left\{f\left(x_{n}(i-1)\right)+f\left(x_{n}(i+1)\right)\right\}\\ f(x)=\mu x(1-x) \end{array}\right.$$ (2)

The equation above combines the i-th spatial index, the n-th time index, and a constant ε, which is within the range of (0, 1). The ranges of 3.57 ≤ *μ* ≤ 4, 0 < *x* < 1, and 0 < *f*(*x*) < 1. define the bounds of parameters in Eq (2).

To take advantage of the benefits of more complex systems, Eq (1) can be substituted into Eq (2). By doing so, a hybrid spatiotemporal htperchaotic model can be obtained as the following equation:

$$x_{n+1}=(1-\varepsilon )f\left(x_{n}(i)\right)+\frac{\varepsilon }{2}\left\{f\left(x_{n}(i-1)\right)+f\left(x_{n}(i+1)\right)\right\},$$ (3)

$$f\left(x_{n}\right)=1-\alpha x_{n}^{2}+y_{n}$$

$$y_{n}=\beta x_{n-1}$$

In the above equation, *f*(*x*) represents a nonlinear hyperchaotic function in Eq (1). The range of variations of the proposed chaotic system is shown in Fig 2 for use in encrypting data.

**Fig 2:** The variation domain of the proposed two-way hyperchaotic system.

As shown in Fig 2, the proposed chaotic system can exhibit chaotic behavior in both dimensions of space and time. On the other hand, considering a new highly sensitive key in this model has eliminated the limitations of the previous model, making it a useful tool for encrypting data.

### 3–2. Proposed encryption algorithm

The proposed encryption algorithm performs data encryption through two phases of confusion and diffusion. The confusion phase involves permuting the data based on a pseudo-random pattern created from the values in the proposed chaotic sequence. Additionally, the diffusion process changes the values of the data. To accomplish this, a rule-based model has been used, which makes it difficult to detect the pattern of data modifications. It should be noted that the proposed algorithm is capable of encrypting any type of data at the byte level, including images, text, and even audio signals. The steps of encryption process in the proposed method is illustrated in Fig 3.

RETRACTED

**Fig 3:** Flowchart of encryption steps in the proposed method.

Without loss of generality, we will explain the encryption steps for two-dimensional (2D) images in the following. For this purpose, we consider an image such as I, with dimensions of *N* = *w* × *h* pixels. In this case, the proposed algorithm for encrypting image I includes the following steps:

**Step 1:** Image *I*_*w*×*h*_ is converted to a vector structured as:*I* = {*i*_1_, *i*_2_, …, *i*_*N*_}.
**Step 2:** The first diffusion stage is performed using the bitwise XOR operator on the image:

$$\left\{\begin{array}{l} i_{1}^{\prime }=i_{1}⊕i_{N}\\ i_{v+1}^{\prime }=i_{v+1}⊕i_{v}^{\prime },\;v=1,\ldots ,N \end{array}\right.$$ (4)

By applying the above equation to the initial vector I, a diffused vector $I^{\prime }=\left\{i_{1}^{\prime },i_{2}^{\prime },\ldots ,i_{N}^{\prime }\right\}$ will be obtained, which will be used as the input for the next step.

**Step 3:** To generate the initial value *x*_1_, the values of the sequence $I^{\prime }$ are multiplied together, and then the resulting value is sequentially divided by 10 to obtain a number within the range [0,1]. The obtained value is used as *x*_1_ in Eq (3). After determining *x*_1_, the sequence *x*_*n*_ is generated based on the proposed hyperchaotic system. This sequence can have a length of 2N, but to cope with the destructing effect of transfer in function, the first T terms of the sequence are neglected. Therefore, from the sequence X with a length of 2*N* + *T*, elements *T* + 1 to *T* + *N* are extracted as a numerical vector like $X^{\prime }=\left\{x_{T+1},x_{T+2},\ldots ,x_{T+N}\right\}$.
**Step 4:** In this step, confusion of pixels is performed on the image. To do this, the values of the X sequence are sorted in descending order, and the order of value permutation in the X’ sequence is generated as a permutation sequence like *P* = {*p*_*ix*(1)_, …, *p*_*ix*(*N*)_}. In this sequence, *p*_*ix*(1)_ represents the index of the element that had the highest value in X’ and has moved to the beginning of the sequence after sorting. Thus, based on the permutation sequence P, the values of the I’ sequence are permuted. By doing so, the permuted data are described in the form of a vector like $I^{\prime \prime }=\left\{i_{ix(1)}^{\prime },\ldots ,i_{ix(N)}^{\prime }\right\}$.
**Step 5:** The next N elements of the X sequence (which was formed in step 3) are organized in the form of a vector like *U* = {*x*_*T*+*N*+1_,*x*_*T*+*N*+2_, …, *x*_*T*+2*N*_}, and based on that vector, Y is created as follows:

$$y_{i}=\lfloor \left(u_{i}\times 10^{20}\right)mod256\rfloor$$ (5)

Using the modulus operator ensures that the values of sequence Y are always within the range [0, 255]. Then, using the vector Y, the second stage of diffusion is applied to the permuted data sequence using the following equation:

$$D_{i}=I_{i}^{"}⊕y_{i}$$ (6)

The vector D, obtained by applying the above equation, is the encoded data after an initial diffusion (step 2), a confusion (step 4), and a secondary diffusion step (step 5). This vector is used as input for the next step.

RETRACTED

**Step 6:** In this step, the final diffusion is performed on the data obtained from the previous step to obtain the encryption result. The proposed method uses a reversible rule-based model, in which each member of the D sequence is changed based on its current and previous values and its neighbors. This process is done using the XOR operator at the bit level. For this purpose, first, based on the chaotic sequence U, a binary sequence like Z is created as follows:

$$z_{i}=\lfloor \left(u_{i}\times 10^{20}\right)mod2\rfloor$$ (7)

The sequence is considered as the previous state of the elements of sequence D. Thus, each member of set D has a current value and a previous value. According to the vector form of D, each element has a left neighbor and a right neighbor (except for the first and last elements of the sequence, which are ignored in this process). In the following, the value of the i-th element of vector D is represented as $d_{i}^{t}$. Thus, $d_{i}^{t-1}$represents the value of the i-th element of D in the previous iteration. Also, the current value of its left neighbor is represented as $d_{i-1}^{t}$. With these explanations, for each bit value in sequence D, a tuple like $<d_{i-1}^{t},d_{i}^{t},d_{i+1}^{t}>$ is formed, and with considering the current value of that bit (i.e. $d_{i}^{t-1}$), the next value $d_{i}^{t+1}$ is determined. The rules for determining the next state of each bit in the proposed method are listed in Table 1.

**Table 1:** The rules defined in the proposed method for determining the next state of each bit.

$d_{i-1}^{t},d_{i}^{t},d_{i+1}^{t}$	$d_{i}^{t+1}$		$d_{i-1}^{t},d_{i}^{t},d_{i+1}^{t}$	$d_{i}^{t+1}$	
	$d_{i}^{t-1}=0$	$d_{i}^{t-1}=1$		$d_{i}^{t-1}=0$	$d_{i}^{t-1}=1$
000	1	0	100	1	0
001	1	0	101	0	1
010	0	1	110	1	0
011	0	1	111	0	1

Based on Table 1, the proposed method changes the value of each bit in the elements of sequence D using 16 rules. For example, if the tuple $<d_{i-1}^{t},d_{i}^{t},d_{i+1}^{t}>$ for a bit has the values of 000, then the previous bit value is checked. If this value is zero $d_{i}^{t-1}=0$, then the new value of the target bit will be 1 ($d_{i}^{t+1}=1$) and otherwise, the value remains zero. According to the described process, in this step, each element in vector D performs the operation of changing the values of its bits for each of its bits based on the rules in Table 1. This operation is repeated *R* times. The result of this operation will be a vector such as $C=\left\{d_{1}^{t+r},\ldots ,d_{N}^{t+r}\right\}$

**Step 7:** Vector C is transformed into a matrix with the same dimensions as the initial matrix I. The matrix *C*_*w*×*l*_ along with the key values used for encryption are considered as the output of the proposed algorithm.

RETRACTED

The encryption steps of the proposed algorithm on a hypothetical 5x5 matrix are shown in Fig 4. It should be noted that for clearer visualization of the encryption steps in the proposed method, the results of applying all the steps on the input are displayed in matrix form. The input to the encryption algorithm is shown in Fig 4A. The result of the initial diffusion (step 2 of the proposed method) is shown in Fig 4B. By multiplying the values in Fig 4B and sequentially dividing by 10, a value of 0.35 is obtained, which is used as the initial value x_1_ in Eq (3), and based on that, the hyperchaotic sequence X is obtained. After sorting the first 25 elements of this sequence, a permutation sequence is created, which, when applied to Fig 4B, results in Fig 4C. The result of the second diffusion step is shown in Fig 4D. Finally, by changing the bit values of the sequence corresponding to this figure using the proposed rule-based model, Fig 4E is obtained, which is the encryption result.

**Fig 4:** Steps of the proposed encryption algorithm on a hypothetical 5x5 matrix.

As the comparison between Fig 4A and 4E shows, the visual pattern in the original image cannot be extracted. In the next section, the performance of the proposed method in data encryption will be thoroughly studied.

### 3–3. Decryption in the proposed method

Data encrypted by the proposed method can be decrypted by performing the inverse processes used for encryption. Thus, having the secret key values, the generated chaotic map and steps 8 to 1 are applied inversely to the encrypted data. Additionally, if the data to be encrypted/decrypted is of the color image type, each of the explained steps will be applied separately to the color layers of the image.

## 4. Results and discussion

The proposed method was implemented using MATLAB 2018a software. During the experiments, the efficiency of the proposed method was evaluated in terms of various aspects of data encryption and the results were compared with similar previous methods. All of the experiments were executed on a personal computer, running 64-bit version of Microsoft Windows 10 on an Intel core i7 3.2 GHz and 8 GB of RAM. During the experiments, the efficiency of the proposed encryption algorithm was evaluated using 10 grayscale and 10 RGB images. The dimensions of input images are different with minimum size of 256 × 256. Also, 10 text documents containing English characters were utilized for evaluating the performance of proposed method in text encryption. Each text document contains at least 12K characters of ASCII table. Finally, 10 audio signals with minimum length of 13 seconds at 96 kbps bitrate were utilized for evaluating the performance of the proposed method in encrypting audio files. In order to better represent the performance of the proposed method, the results presented in this section are based on the encryption of image data. In this regard, results for encrypting four mostly-used images in this field are presented, including: cameraman and Lena images in grayscale color system; and mandrill and peppers images in RGB color system.

RETRACTED

### 4–1. Visual and histogram analysis

First, the efficiency of the proposed method in encrypting information is examined based on visual results and histogram analysis. To this end, images with different color systems are encrypted and then decrypted, and the changes in the images and their histograms during this process are examined. Fig 5 shows the encryption and decryption results for the "camera" image. In this figure, the original image is shown on the left, the encryption result is shown in the middle, and the decryption result is drawn on the right. Additionally, for each state, the image is shown at the top and its histogram is shown below it.

**Fig 5:** The camera image and its histogram after encryption and decryption.

Since the camera image is in grayscale, the encryption process only applies to the single layer of the image. By examining the results presented in Fig 5, several important conclusions can be reached. Firstly, none of the patterns present in the original image are visible in the encrypted result. This feature indicates that visual inspection of encrypted information cannot lead to any insights regarding the secret content. Secondly, the decrypted image has a minimum difference with the original image. Thus, the proposed encryption algorithm imposes minimal changes on the input data. The comparison of the histograms of the input and decrypted images confirms this claim. On the other hand, by comparing the histograms of the input image with the encrypted image, it can be seen that the proposed method changes the intensity values of the pixels in a way that the encryption result looks like a matrix with random values. This feature is achieved in the proposed method through three stages of diffusion, allowing for pixel values to be altered in a way that does not have any recognizable relationship with the original data. The uniformity of the encrypted image indicates its efficiency in resistance against statistical attacks. In Fig 6, the same results are shown for the chilies image.

RETRACTED

**Fig 6:** The chilies image and its histogram after encryption and decryption.

As the chilies image has an RGB color system, similar to the process described in the previous section, encryption operations are performed separately on each color layer. The results presented in this figure confirm that the proposed method for encrypting color images also performs well, as the histograms of the encrypted color layers are uniform and no information can be extracted about the color changes in the original image. The encryption and decryption results for hummingbird and baboon images are shown in Figs 7 and 8, respectively.

**Fig 7:** Hummingbird image and its histogram after encryption and decryption.

**Fig 8:** Baboon image and its histogram after encryption and decryption.

To further investigate the resistance of the proposed method against statistical attacks, the standard deviation measure of the frequency values in the histogram of the encrypted image can be used. Therefore, the standard deviation measure is calculated for the number of pixels with different brightness intensity values in the encrypted image. In color images, this operation has been performed separately for each color layer. The results of this analysis are presented in Table 2. As shown in Table 2, the proposed method can encrypt images in a way that results in images with a more uniform brightness and no visible pattern. These results indicate that the proposed method can perform better against statistical attacks compared to the other methods.

**Table 2:** Standard deviation of frequency values in the histograms of encrypted images.

	Cameraman	Peppers	Lena	Mandrill	Average
**Proposed Method**	15.9625	28.3336	31.3165	16.6375	23.0625
**Zhang et al [20]**	17.5628	29.1999	34.5682	18.1756	24.8766
**Alexan et al [24]**	16.8585	28.8524	34.8889	16.3515	24.2378
**Hosny et al [22]**	19.5625	28.6548	35.5556	17.8890	25.4155
**Abduljabbar et al [25]**	-	32.5645	37.1865	19.5685	29.7732

### 4–2. Analysis of correlation in adjacent pixels

Correlation analysis is used to find the similarity between the bytes of the original data and the encrypted data. In an image, neighboring byte values in the original data are strongly correlated in three directions: horizontal, diagonal, and vertical. An efficient encryption method is one that reduces this correlation in the encrypted data. The correlation coefficient value is in the range [–1, 1], and its value for the encrypted data should be close to 0. To analyze the correlation, first, 1000 random pairs of neighboring pixels that can have one of the horizontal, vertical, or diagonal neighbor states are selected from the original image, and their correlation is calculated. Then, the correlation level is calculated for the same pixels in the encrypted image. The correlation measure is calculated using the following equation [28]:

$$r_{xy}=\frac{\mathrm{cov}(x,y)}{\sqrt{D(x).D(y)}}$$ (8)

Which in the above equation, we have [28]:

$$cov(x,y)=\frac{1}{N}\overset{}{\underset{}{\sum_{i=1}^{N}\left(x_{i}-\bar{x}\right)\left(y_{i}-\bar{y}\right)}}$$ (9)

And [28]:

$$D(x)=\frac{1}{N}\sum_{i=1}^{N}{\left(x_{i}-\bar{x}\right)}^{2}$$ (10)

In the above equations, x_i_ and y_i_ represent the values of neighboring pixels. The correlation analysis results for the cameraman image are shown in the form of graphs in Fig 9. Also, in Fig 10, the same results are presented for the peppers image.

RETRACTED

**Fig 9:** Correlation analysis results for the cameraman image.

**Fig 10:** Correlation analysis results for the peppers image.

In Figs 9 and 10, correlation plots of neighboring pixel intensities for the original image are displayed in the first row, while the second row shows the results for the encrypted image. Additionally, the horizontal, vertical, and diagonal correlations for each case are shown in the left, middle, and right columns of these figures, respectively. Based on Figs 9 and 10, the original images exhibit high correlation values among neighboring pixels, visible in various directions. This is because the correlation plots for input images are formed around x = y axis, meaning that for each pixel with value x in the original image, its neighboring pixels will have similar values (*x* ≅ *y*). In contrast, the correlation of neighboring pixel values in encrypted images does not exhibit any pattern, and correlation points are scattered throughout the plot. The numerical values obtained from the correlation test are given in Table 3.

**Table 3:** Numeric values obtained from the correlation analysis of adjacent pixels.

	Proposed Method	Zhang et al [20]	Alexan et al [24]	Hosny et al [22]	Abduljabbar et al [25]
**Lena**					
horizontal	0.00114	-0.0029	0.00144	0.00414	0.0033
diagonal	0.00801	-0.0021	-0.00151	-0.00792	0.0027
vertical	0.00421	0.0049	0.00795	0.00533	0.0070
**Camera Man**					
horizontal	-0.00107	0.0002	0.00566	0.00145	-
diagonal	0.00072	-0.0034	0.00078	0.00156	-
vertical	0.00077	-0.0020	0.00574	0.00178	-
**Peppers**					
horizontal	0.00020	0.0018	-0.00021	0.00218	-0.0020
diagonal	-0.00028	0.0027	0.00027	0.00087	-0.0064
vertical	0.00103	0.0016	0.00128	0.00199	0.00008
**Mandrill**					
horizontal	0.00011	0.0019	0.00004	-0.00079	0.0025
diagonal	-0.00016	-0.0013	-0.00021	0.00056	0.0035
vertical	0.00024	0.0030	0.00039	0.00044	0.0064
**Average**	**0.0015**	**0.0023**	**0.0021**	**0.0024**	**0.0037**

Based on the results presented in Table 3, the proposed method can encrypt images in a way that leads to lower average correlation. This indicates the superiority of the proposed method in maintaining information security, which can be attributed to the use of the proposed confusion and multi-stage diffusion strategies. Therefore, extracting patterns of sensitive data through encrypted images in the proposed method will be more difficult.

RETRACTED

### 4-3- Analysis of the difference between the original and encrypted data

The purpose of this test is to examine the performance of the proposed encryption algorithm in creating data that is different from the original information. To do this, the input data is first encrypted based on the proposed encryption strategy, and then the encrypted information is compared with the original data. For this purpose, two criteria, Mean Squared Error (MSE) and Bit Error Rate (BER), are used. The MSE criterion measures the difference between the encrypted values and the original data at the byte level, while using the BER criterion, this difference can be measured at the bit level. The MSE criterion can be calculated based on the following equation [29]:

$$MSE=\frac{1}{N}\overset{}{\underset{}{\sum_{i=1}^{N}{\left[O(i)-R(i)\right]}^{2}}}$$ (11)

In the above equation, i represents the byte position of the data and N represents the number of data bytes. O refers to the original data and R represents the encrypted data. The MSE value is in the range of [0, ∞] and the desirable state is to maximize the MSE value between the original and encrypted data. In contrast, the BER criterion can be calculated as follows [29]:

$$BER=\frac{\sum_{i=1}^{N}O(i)⊕R(i)}{N}$$ (12)

In the above equation, i represents the position of a data byte, and N is the total number of data bytes. O refers to the original data, and R represents the encoded data. The symbol ⨁ denotes the XOR operation. The BER value ranges from 0 to 1, and the desirable state for an encryption algorithm is to maximize the BER between the original and encoded data. Fig 11 compares the average BER and MSE of the proposed method with other methods for encrypting various types of data.

RETRACTED

**Fig 11:** Comparison of the performance of the proposed method with other methods in terms of (a) MSE and (b) BER metrics.

Based on the results presented in Fig 11, the MSE and BER values between the original data and the encryption result in the proposed method are higher than the compared methods. Therefore, the encrypted data by the proposed method have a greater difference with the details of the original data. These results indicate that the proposed method can increase the MSE metric by at least 14.15% and the BER metric by at least 1.79% (compared to the closest performing method to the proposed method, Alexan et al. [24]).

### 4–4. Analysis of key sensitivity and key space

High sensitivity of the key and availability of a wide space for selecting authorized keys in an encryption algorithm increases its resistance against Brute-Force attacks. The sensitivity of the key refers to the smallest change in the key values that leads to a change in the encryption or decryption result. The proposed algorithm uses three primary keys, α, β, and ε, for data encryption. The smallest effective change on the chaotic sequence for keys α and β is equal to 10^-10^. On the other hand, the sensitivity of key ε in the proposed chaotic system is equal to 10^-28^. The key selection space for α and β is 0.5, while key ε can have values in the range of (0,1) to show chaotic behavior. Therefore, the number of valid combinations for selecting keys in the proposed method will be equal to 10^38^. In this case, if a computer with high processing power is able to test one billion combinations per second, then checking all possible cases to obtain valid keys through Brute-Force attacks will take more than 3.17 × 10^21^years. Thus, it can be concluded that the high key space and their sensitivity in the proposed method will make it secure against Brute-Force attacks. Fig 12 shows the effect of changes in each of the keys on the chaotic sequence. As shown in this figure, making partial changes to each of the keys in the proposed method can cause overall changes in the generated sequence. These changes will affect the patterns of confusion and diffusion in the encryption process. This suitable performance can be attributed to the use of the proposed hybrid hyperchaotic model.

**Fig 12:** The effect of changes in (a) α, (b) β, and (c) ε on the chaotic sequence generated in the spatial domain.

### 4–5. Entropy test

Information entropy is a well-known and widely used measure for assessing the randomness of information, which is extensively used for evaluating the quality of encryption. This measure can be calculated as follows [30]:

$$H(m)=-\sum_{i=1}^{2^{n}-1}p\left(m_{i}\right)\log_{2}\frac{1}{p\left(m_{i}\right)}$$ (13)

Where, m represents the information being evaluated and *p*(*m*_*i*_) describes the probability of the presence of data *m*_*i*_ in this information. In information organized by bytes (such as text characters or grayscale image pixels), the ideal random state has an entropy of 8. Therefore, in an encryption system that encrypts information at the byte level, the encrypted data should have an entropy close to 8. Table 4 shows the results of the entropy test on various image, text, and audio data types. Also, the results of the proposed method are compared with other methods. In this table, the results of proposed method have also been compared with AES [31] and DES [32] algorithms to cover all types of data for encryption.

RETRACTED

**Table 4:** Results of entropy testing on various types of image, text, and audio data for the proposed method.

	Grayscale Images	RGB Images	Text Data	Audio Data
**Proposed Method**	7.9994	7.9992	7.9992	7.9995
**Zhang et al [20]**	7.9991	7.9995	-	-
**Alexan et al [24]**	7.9987	7.9968	-	-
**Hosny et al [22]**	7.9981	7.9976	-	-
**Abduljabbar et al [25]**	7.9990	7.9991	-	-
**AES [31]**	7.9972	7.9968	7.9961	7.9977
**DES [32]**	7.9969	7.9959	7.9960	7.9973

Since the methods presented in [20, 22, 24, 25] are proposed for encrypting image data, there is no information available on their ability to encrypt textual and audio data. Based on the results presented in Table 4, the encrypted data by the proposed method has a high entropy close to 8, independent of the data type being encrypted. The higher entropy of the proposed method compared to other methods indicates its higher efficiency in the processes of confusion and diffusion. Therefore, the proposed solution can be effective in enhancing the security of encrypted data.

### 4–6. Time analysis

In this experiment, the performance of the proposed method in term of processing time has been evaluated. For this purpose, the processing time for encryption and decryption operations of the proposed method has been compared with previous works. These results are presented in Table 5. These results are obtained through calculating the average processing time of encrypting/decrypting 10 colored images with size of 256 × 256. It should be noted that the reported processing times are obtained through machines with different specifications, which are listed in Table 5.

**Table 5:** The average processing time of encrypting/decrypting colored images.

Methods	Encryption time (s)	Decryption time (s)	Machine Specs (CPU, RAM)
**Proposed Method (R = 1)**	0.30564	0.32565	(3.2 GHz intel core i7, 8GB)
**Proposed Method (R = 2)**	0.51156	0.53765	(3.2 GHz intel core i7, 8GB)
**Proposed Method (R = 3)**	0.71690	0.77026	(3.2 GHz intel core i7, 8GB)
**Zhang et al [20]**	3.77630	-	(1.8 GHz intel core i5, 8GB)
**Alexan et al [24]**	2.75096	-	(3.4 GHz inter core i7, 8GB)
**Hosny et al [22]**	1.56801	1.89500	N/A
**Abduljabbar et al [25]**	0.34940	0.41670	N/A

In Table 5, the processing time of proposed method has been examined for *R* = {1, 2, 3}; which R refers to the number of cycles for applying final diffusion on image bits using reversible rule sets. It should be noted that, during all of the previous experiments, this parameter was considered as *R* = 2. It is obvious that increasing the number of cycles lead to more processing time for encryption and decryption operations. However, by increasing the value of R, the proposed method can still compete with other methods in terms of processing speed. These results confirm the proper performance of the proposed method for fast data encryption.

RETRACTED

Table 6, lists the summary of the results obtained through experiments of the research. In this table, the average values of different metrics in addition to average improvement obtained by the proposed method is presented. Also, the best result of each experiment is bolded in the table.

**Table 6:** Summary of the results obtained through experiments of the research.

Metrics	Proposed Method	Zhang et al [20]	Alexan et al [24]	Hosny et al [22]	Abduljabbar et al [25]	Average Improvement (%)
**Correlation**	**0.0015**	0.0023	0.0021	0.0024	0.0037	40.07% ↓
**MSE**	**10413**	8945.6	9122.1	9004.5	-	15.39% ↑
**BER**	**0.4999**	0.4855	0.4911	0.4892	-	2.315% ↑
**Entropy**	**7.9993**	**7.9993**	7.9977	7.9978	7.99905	0.010% ↑
**Processing Time**	0.5246	3.77630	2.75096	1.7315	**0.3831**	49.95% ↓

According to the summary of the results presented in Table 6, the overall efficiency of the proposed method is better than the compared studies. The results showed that the proposed method needs more processing time compared to the work by Abduljabbar et al [26]; but has superiority in other aspects. As shown in Table 5, this increased processing time comes from the final rule-based diffusion step of the proposed method which can be addressed in future works.

## 5. Conclusion

In this article, a new method for data encryption using hyperchaotic system was proposed. In this study, a highly sensitive hyperchaotic model with a wider key space was presented to overcome the shortcomings of previous models. The proposed encryption strategy is based on the diffusion and confusion strategy. The performance of the proposed method in encrypting various types of data has been studied and the results have been compared with previous solutions. The results of visual and histogram analysis show that the proposed method can change the values of encrypted data in a way that a uniform histogram with minimum standard deviation is obtained. This, makes the proposed method to provide a high resistance against statistical attacks. The results of correlation analysis indicate a significant reduction in correlation between neighboring data by the proposed encryption algorithm; which is at least 28.57% less than previous works. Therefore, the proposed method may make it impossible to detect and analyze patterns between encrypted data to obtain primary information. Based on the results of the analysis of the difference between the initial data and the encrypted data, the proposed method increases the MSE and BER metrics by at least 14.15% and 1.79%, respectively; which indicate that the data encrypted by the proposed method have a greater difference with the details of the initial data. Also, the large key space and high sensitivity to changes in key values in the proposed method make it resistant to brute-force attacks. The proposed method encrypts data with higher entropy which is independent of the type of data. This is evidence of its higher efficiency in the confusion and diffusion processes compared to other methods.

RETRACTED

One of the limitations of the proposed method is its longer computational time for the final diffusion step, which is performed using a reversible rule-based model. In future work, it is possible to reduce this processing time by optimizing this mechanism and using parallel computing techniques.

## Supporting information

S1 Dataset (ZIP)
